The article "Comparing Thoracic Extensive Laminoplasty (TELP) and Laminectomy in Treating Severe Thoracic Ligamentum Flavum Ossification: A Proposed Novel Technique and Case-Control Study" was published in 2021. Journal: Biomed Res Int.

# Comparing Thoracic Extensive Laminoplasty (TELP) and Laminectomy in Treating Severe Thoracic Ligamentum Flavum Ossification: A Proposed Novel Technique and Case-Control Study

**DOI:** 10.1155/2021/8410317

**Published:** 2021-04-20

**Authors:** Jun Ma, Zhengyu Lu, Xin Zhou, Jia Yin, Enjie Xu, Heng Jiang, Xiao Ma, Yichen Meng, Zhilin Li, Rui Gao, Tao Lin, Xuhui Zhou

**Affiliations:** ^1^Department of Orthopedics, Changzheng Hospital, Second Affiliated Hospital of Second Military Medical University, 415 Fengyang Road, Shanghai, China 200003; ^2^Department of Advertising, School of Journalism, Fudan University, 220 Handan Road, Shanghai, China 200000

## Abstract

**Objective:**

(1) To propose a novel technique named thoracic extensive laminoplasty (TELP) in curing severe thoracic ligamentum flavum ossification (STOLF) and (2) to compare outcomes between TELP and laminectomy in curing STOLF.

**Methods:**

Cases with fused or tuberous STOLF (Sato classification) treated from Jan 2015 to Jan 2017 were reviewed and divided into the TELP group (G1) and laminectomy group (G2) according to their surgical management. Data on demographics, complications, pre- and postoperative symptoms, residual spinal canal area (RSCA-1), residual spinal cord area (RSCA-2), modified Japanese Orthopedic Association score (mJOA), and health-related quality of life (HRQOL, based on the SF-36) were collected.

**Results:**

Fifty-nine G1 and sixty-two G2 patients were enrolled. No significant differences in demographic data or preoperative data of RSCA-1, RSCA-2, mJOA, or HRQOL were observed between the two groups (*p* > 0.05). Patients in G1 and G2 showed similar postoperative improvements in RSCA-1 and RSCA-2 at the final follow-up (*p* > 0.05). However, patients in G1 showed higher postoperative improvements in mJOA (OR = 2.706, 95% CI: 1.279~5.727, *p* = 0.008) at the final follow-up. Patients in G1 also showed higher postoperative improvements in HRQOL than patients in G2 (*p* < 0.05) at the final follow-up, and patients with more severe STOLF presented with better improvements in HRQOL in G1 (*p* < 0.05). Dural laceration and cerebrospinal fluid leakage were observed in seven G2 patients, and no complications were found in G1 patients after surgery.

**Conclusion:**

TELP is a novel, effective, and safer surgical technique in treating STOLF and could be a substitute for traditional laminectomy.

## 1. Introduction

Thoracic ossification of the ligamentum flavum (TOLF) is the most common cause of thoracic spinal stenosis, and it eventually leads to thoracic myelopathy, which was first reported by Tamaguchi et al. in 1960 [1]. TOLF occurs mainly in East Asia, including Korea, Japan, and China. Previous studies indicated that the incidence of TOLF was 21.8% (1090/4999) [2], 12% (180/1500) [3], and 3.8% (66/1736) [4] in Korea, Japan, and China, respectively. In China, it was reported that 63.9% of patients with chest symptoms were diagnosed with TOLF [5]. Meanwhile, the onset and progression of TOLF are insidious and chronic, which causes the diagnosis to frequently be missed and delayed. Most patients have already had a loss of functional gait when they come to see a doctor, and their prognosis is always poor [6, 7]. Thus, how to effectively treat TOLF (especially severe TOLF (STOLF)) is still a challenge for doctors.

Sato et al. classified TOLF into five types according to its severity, and the fused and tuberous types were the most severe disorders. For STOLF, surgical management is the only effective treatment option [8, 9]. Laminectomy is the traditional and currently recommended method for treating STOLF. The incidence of dural ossification in patients with STOLF is 43.4% [10], and complications of dural laceration and cerebrospinal fluid leakage are quite common during laminectomy, affecting approximately 10-32% of cases in a previous study [11]. Laminectomy combined with patch grafting is suggested for the treatment of STOLF with iatrogenic dural laceration, and laminectomy combined with floating the ossified dura by thinning it with a drill is applied for treating STOLF while avoiding damage to the dura. Both methods were thought to be effective in previous studies with a small sample size [12, 13]; however, considerations of infection, neurological damage, and operative complexity cannot be ignored. Thus, searching for a more effective and safer surgical method for the treatment of STOLF is of great value.

In our study, we aimed (1) to propose a novel surgical technique named thoracic extensive laminoplasty (TELP) for curing STOLF and (2) to verify the superior efficacy of TELP compared with traditional laminectomy (LT).

## 2. Materials and Methods

Cases of TOLF from Jan 2015 to Jan 2017 were reviewed in our hospital, and a case-controlled study was conducted. All patients were classified into two groups based on the surgical procedures they received: (1) patients who received TELP were grouped into G1, and (2) patients who received LT were grouped into G2.

### 2.1. Inclusion Criteria

Inclusion criteria are as follows:

1. Age from 40 to 60 years old
2. Followed up for at least 18 months
3. Complete preoperative and postoperative anteroposterior thoracic plain X-ray, CT, and MRI
4. Complete preoperative and postoperative evaluation of the modified Japanese Orthopedic Association score (mJOA) and health-related quality of life (HRQOL, based on the SF-36)
5. All patients had fused or tuberous-type (Sato classification) TOLF, which was considered severe TOLF (STOLF).

### 2.2. Exclusion Criteria

1. Patients with articular diseases of the axial skeleton, traumatic fractures of the spine, thoracic intervertebral disc herniation, and other ossifications of the spinal ligamentum were excluded
2. Patients with cervical, lumbar, and sacral diseases were excluded
3. Patients with diseases that influenced bone healing, such as osteoporosis, multiple myeloma, bone cancer, and bone tuberculosis, were also excluded.

### 2.3. Evaluation of Demographic Characteristics

Data on age, sex, body mass index (BMI), symptoms, blood loss, operating room time, follow-up time, postoperative dural laceration, and cerebrospinal fluid leakage (CSFL) were collected.

### 2.4. Image Evaluation

Patients with more than 50% levels of tuberous TOLF were considered to have the tuberous type (T), and patients with more than 50% levels of fused TOLF were considered to have the fused type (F). Levels of STOLF, dural ossification or dural adhesion (comma sign or track sign), preoperative and postoperative residual spinal canal area (RSCA-1), and residual spinal cord area (RSCA-2) were evaluated based on CT and MRI.

The measurement method was performed according to Liu et al. [1] and is shown in Figure 1. If patients had more than one level of STOLF, we calculated the mean RSCA-1 (or RSCA-2) of all of the levels as the final result. The calculation of improvement was as follows: postoperative RSCA − 1 (or RSCA − 2)–preoperative RSCA − 1 (or RSCA − 2).

### 2.5. Neurological Evaluation

mJOA was collected before and after surgery or neurological assessment. The Hirabayashi recovery rate was calculated as follows [14]: recovery rate = (postoperative JOA score − preoperative JOA score)/(11 − preoperative JOA score) × 100%.

### 2.6. Health-Related Quality of Life (HRQOL) Evaluation

HRQOL was evaluated before and after surgery based on the SF-36. Sections of physical functioning (PF), bodily pain (BP), general health (GH), and reported health transition (RHT) were included. The survey was in Chinese, and the normalized score was calculated according to Li et al. [15]. Normalized score = (Actual score–The lowest score of the section)/(The highest score of the section–The lowest score of the section) × 100. Based on the calculated normalized score, the recovery rate was calculated as follows: recovery rate = (postoperative section score − preoperative section score)/(100 − preoperative section score) × 100%. The lowest score of the section means the lowest score that patients can acquire in this section. The highest score of the section means the highest score that the patient can acquire in this section.

### 2.7. Statistical Analysis

We adopted the SPSS statistical analysis software version 13.0 (SPSS, Inc., Chicago, IL) for evaluation. Quantitative data were analyzed by Student's *t*-test, and classic data were analyzed by the Wilcoxon signed-rank test. Chi-squared analysis was also performed. Differences were considered significant when the *p* value < 0.05.

### 2.8. Ethics Statements

This research project was approved by the ethics department of our hospital. We obtained consent from all participants. All procedures were performed under the principles of the Declaration of Helsinki and relevant policies in China.

## 3. Results

### 3.1. Surgical Procedure of TELP

Endotracheal anesthesia was performed, and the patient was placed in the prone position before surgery. Neurophysiological monitoring involving somatosensory evoked potentials (SSEPs) and motor-evoked potentials (MEPs) was conducted throughout the entire process. A C-arm X-ray machine was used to target the influenced levels of the thoracic vertebrae pre- and intraoperatively. A posterior midline longitudinal incision was made, and procedures were adopted to completely expose the spinous processes, bilateral lamina, bilateral zygapophyseal joints, and the bilateral transverse process of the influenced levels. Tissues of the involved levels, including the spinous process, inferior portions of the superior lamina, superior portions of the inferior lamina, and interlamina ligamentum flavum, should be excised gently. Then, the normal boundaries of the thoracic spinal cord needed to be confirmed. Along the bilateral connections of the midpoint of the facet joints, which were taken as references, grinding was performed with a drill (Stryker, 4.0 mm) at the lamina bilaterally. When the inner cortical bone was exposed, holes were drilled for the following fixation of the arch plate at the transverse process and lamina. Then, the grinding procedure was continued (Stryker, 3.0 mm) until the lamina was isolated. Bipolar electrocoagulation and sterilized medical bone wax were used for hemostasis throughout the operation.

The connections of the soft tissues of the lamina were separated with a hooker nerve stripper from the caudal direction to the cephalad direction along the surface of the dural sac. Then, the arch plates were fixed bilaterally. Posterior fusion was carried out at the bilateral transverse process and the lamina with corticocancellous bone. To adjust the narrow part, an O-arm X-ray machine was used for space assessment of the spinal canal during the operation. All of the operative procedures are illustrated in Figures 2 and 3.

### 3.2. Surgical and Clinical Outcomes

A total of 59 patients in G1 (Figure 4) and 62 patients in G2 (Figure 5) were enrolled, and no patients were lost to follow-up. The average follow-up times were 19.4 ± 2.1 months and 18.9 ± 2.8 months in G1 and G2, respectively, and no significant differences were observed (*p* = 0.271). The average age, BMI, and sex proportions were similar between G1 and G2 (*p* > 0.05). In G1, the number of patients with lower limb (LB) numbness, LB spastic paraparesis, LB sensory deficits, gait instability, and urinary sphincter dysfunction was 42, 28, 49, 26, and 18, respectively. In G2, 46, 33, 51, 29, and 22 patients had LB numbness, LB spastic paraparesis, LB sensory deficits, gait instability, and urinary sphincter dysfunction, respectively. No significant constitutional differences were observed between G1 and G2 (*p* > 0.05). The average blood loss was 273.8 ± 31.7 ml in G1 and 281.4 ± 35.8 ml in G2, and no significant differences were observed (*p* = 0.220). There were 7 patients with a dural laceration and 7 patients with cerebrospinal fluid leakage in G2; however, no patients with complications were found in G1 after the surgery (Table 1).

The levels of STOLF had no significant constitutional differences between the two groups (*p* = 0.325). The incidence of dural ossification or dural adhesion was 84.7% (50/59) in G1 and 83.9% (52/62) in STOLF. Significant improvements in RSCA-1 were observed in both G1 (*p* < 0.0001) and G2 (*p* < 0.0001) after surgery, but no significant preoperative or postoperative differences in RSCA-1 were found between G1 and G2 (*p* > 0.05). Similar results were also found when we evaluated RSCA-2 (Table 2).

The average mJOA was 4.2 ± 1.4 in G1 and 4.3 ± 1.7 in G2, and no significant differences were found (*p* = 0.725) before surgery. The mean postoperative mJOA was 8.1 ± 1.9 in G1 and 7.9 ± 1.6 in G2, and no significant differences were found (*p* = 0.532). The mJOA of patients in G1 and G2 all improved significantly (*p* < 0.05) after surgery. However, G1 had better neurological improvements (≥50% recovery rate of mJOA) than G2 (*p* = 0.008, OR =2.706, 95% CI: 1.279~5.727) (Table 3).

HRQOL was also assessed in G1 and G2 (Table 4). The preoperative PF, BP, GH, and RHT of HRQOL in G1 were 31.2 ± 11.4, 52.9 ± 11.7, 37.4 ± 13.9, and 28.9 ± 8.7, respectively, and 31.7 ± 12.1, 53.1 ± 10.8, 37.2 ± 10.7, and 28.2 ± 9.5 in G2, respectively. No significant differences were observed between the two groups (*p* > 0.05). The postoperative PF, BP, GH, and RHT of HRQOL in G1 were 71.6 ± 13.9, 80.6 ± 9.4, 73.4 ± 16.5, and 70.7 ± 11.1, respectively, and 64.8 ± 11.7, 74.3 ± 7.1, 66.2 ± 12.2, and 66.4 ± 10.9 in G2, respectively, and the scores in G1 were higher than those in G2 (*p* < 0.05). The PF, BP, GH, and RHT of the HRQOL of patients in G1 and G2 all improved significantly (*p* < 0.05) after surgery. In G1, tuberous-type patients had better PF improvements (≥50% recovery rate of PF) than fused-type patients (*p* = 0.007, OR = 4.443, 95% CI: 1.471~13.423). Similar results were observed in BP, GH, and RHT of HRQOL. However, this interesting phenomenon was not found in G2.

## 4. Discussion

In our study, we proposed a novel technique of TELP for the treatment of STOLF. We also compared the radiographic, clinical, and HRQOL outcomes between patients who underwent TELP and those who underwent traditional laminectomy. Image evaluation showed that preoperative and postoperative RSCA-1 (or RSCA-2) had no significant differences between G1 and G2 (*p* > 0.05), and both techniques could provide effective and stable decompression of the spinal canal and cord. The average preoperative and postoperative mJOA values were not different between G1 and G2 (*p* > 0.05), and both techniques improved neurological function (*p* < 0.05). However, G1 had a better neurological recovery rate than G2 (*p* = 0.08, OR = 2.706). G1 had better HRQOL (based on the average PF, BP, GH, and RHT scores) than G2 (*p* < 0.05). In addition, G1 patients with more severe types of STOLF (tuberous type) tended to have better rehabilitation of HRQOL (*p* < 0.05); however, this phenomenon was not found in G2 patients.

Symptomatic thoracic myelopathy secondary to TOLF was the indication for surgical intervention, and sufficient decompression of the spinal canal was the key factor influencing the recovery efficacy. TOLF was classified into 5 types based on the severity of the ossified lesion configuration: lateral type, extended type, enlarged type, fused type, and tuberous type. Posterior decompressive surgery was recommended for TOLF, and the laminectomy technique was recommended. It was also suggested that en bloc laminectomy was suitable for the lateral and extended types, and separating laminectomy was ideal for thickening the tuberous type [13].

A previous radiology study also showed that laminectomy could provide significant improvements in canal diameter in curing TOLF (15.1 ± 6.8%, *p* < 0.05) [16]. However, laminectomy has two main inevitable limitations, especially for STOLF. First, dural laceration combined with cerebrospinal fluid leakage, which could lead to cerebrospinal fluid pseudocysts, respiratory obstruction, wound dehiscence, and meningitis, cannot be ignored [17, 18], and dural ossification (DO) or dural adhesion (DA) is the reason for these complications. DO or DA is commonly seen in STOLF, and the reported incidence ranges from 22% to 62% [19–21]. Our data showed that the incidence was 84.7% (50/59) in G1 and 83.9% (52/62) in STOLF. Thus, some researchers have suggested that floating ossified lesions of the dural sac with a high-speed drill to abrade them until paper thin would benefit this situation [22]. However, this results in a lesser extent of spinal decompression, and there is still a high risk of iatrogenic dural tears. Second, laminectomy and excessive resection of the facet joints would cause structural instability, especially for multiple levels of STOLF [23]. It was reported that TOLF is located in multiple segments, tandem ossification is common, and its incidence is 33.3% to 55.1% [24, 25]. Structural instability would cause increased kyphotic deformity of the spine, which would lead to late neurological deterioration. Thus, laminoplasty was proposed. However, laminoplasty was not suitable for STOLF, as this technique could only achieve limited decompression without removal of the ossified ligamentum flavum. Laminectomy with fusion also remains controversial. Therefore, seeking a more effective surgical technique is urgent.

Our study proposed a novel surgical technique for STOLF called TELP. This technique had similar decompressive efficacy as laminectomy (with no significant differences in RSCA-1 and RSCA-2 between G1 and G2). No complications of dural laceration or cerebrospinal fluid leakage were observed, while 7 patients with dural laceration and cerebrospinal fluid leakage were found in the laminectomy group. Increased kyphotic deformity of the spine was not observed in G1 at the final follow-up.

To achieve these goals, the technique has several benefits. First, the isolated lamina could be elevated according to the decompressive demand, which could provide a sufficient volume of spinal canal. In addition, we did not resect the ossified lesions that adhered to the lamina and the dural sac during the procedure. Thus, the suitably and gently lifting force on the lamina would not cause dural tears, and sufficient decompression of the spinal cord would be achieved. Moreover, arch plate placement combined with bone grafting and the residual facet joint reconstructed the posterior column of the spine, which provided sufficient stability to avoid kyphotic deformity of the spine. In addition, the ossified lesion that we did not resect would not cause a second compression, and spontaneous reduction (or atrophy) was observed during the follow-up. Many studies have indicated the same phenomenon, and it is believed that pulsations of the thecal sac and venous plexus are responsible [26–28].

Previous studies demonstrated that the average recovery rate of neurological function based on mJOA was 40% to 50% after laminectomy in TOLF, which indicated fair rehabilitation [29–31]. Our studies also showed similar results for the reported outcomes in G2. No obvious differences in the average preoperative and postoperative mJOA were found between G1 and G2 (*p* > 0.05). Interestingly, we found that the outcome of neurological function in G1 was superior to that in G2 when we compared the number of patients with a ≥50% mJOA recovery rate between G1 and G2. These results indicated that TELP might be more suitable for STOLF than laminectomy, which could be explained by the less invasive procedure of TELP that decreased the risk of neurologic damage. In addition, the spinal cord in the thoracic spine has worse vascularity and occupies a larger proportion of the spinal canal, making it more susceptible to damage by a more invasive procedure [32]. Additional studies are needed for confirmation.

Our study also included an evaluation of the HRQOL of the patients based on the SF-36. To our knowledge, this was the first study to use a patient-reported scale as a part of the assessment of surgical efficacy. For PF, BP, GH, and RHT, both G1 and G2 had significant improvements after surgery, but G1 had better recovery than G2. These results indicated that patients who underwent TELP had better recovery of sensation than those who underwent laminectomy. This was an interesting phenomenon, and we supposed that this could be attributed to the less invasive procedure and no surgical complications in G1. Another interesting phenomenon was that patients with more severe TOLF conditions presented with better recovery of sensation in G1, while this phenomenon was not observed in G2. We supposed that preoperative expectations were the main reason for this phenomenon. Patients with tuberous-type TOLF suffer from more severe symptoms, and a small improvement might provide them with more recovery satisfaction [33]. In addition, TELP is less invasive, and no complications were observed, which might be another reason for this finding. Additional studies are necessary.

Recently, Sun et al. [28] reported a new surgical technique for TOLF that used transverse connectors and surgical lines to build a “bridge crane” to suspend the lamina for the purpose of decompression. The extent of decompression was controlled by the extent of tightening of the surgical lines. This was absolutely an innovation in the surgical community; however, three main limitations should be considered. First, the structural stability was of concern. If the surgical lines are not tightened after adhering to the connector, the isolated lamina attached to the lines will shake, which might cause damage to the dural sac. Actually, the surgical lines could not always be tightened after adhering to the connector because of the consideration of not tearing the dural sac. Second, the surgeon needed to drill a tunnel into the lamina for the surgical line, which was complicated and had a risk of puncturing the dural sac. Finally, the space of the thoracic vertebral canal and pedicle was narrow, and the use of pedicle screws would cause insufficient decompression. In addition, the cost of TELP is lower than that of bridge cranes. Our novel technique of TELP with an arch plate as the fixation material overcame all of the above limitations. Surgeons could control the decompression by changing the angle of the arch plate, which is safe and reliable.

However, several limitations of this study exist. First, the sample size was small, and the follow-up time was limited, which would decrease the reliability and validity of the study. Second, the pulsative movement of the dura mater could not be directly observed, which made intraoperative judgment of decompression of the spinal cord difficult. Third, it was difficult to achieve hemostasis directly, as the structures inside the canal were not visible.

## 5. Conclusion

Our study proposed a novel and effective TELP technique for STOLF. We found that this technique was equivalent to laminectomy in canal and spinal cord decompression. However, our technique was better for neurological recovery, and patients also experienced better HRQOL recovery. TELP could also decrease the risk of dural tears and late-onset kyphotic deformities of the spine, especially for multisegmental STOLF. We hope that our TELP will benefit patients as well as surgeons. Our future research direction will be to conduct a large-scale cohort study for additional evaluation of this technique.

## Figures and Tables

**Figure 1:** Illustration of residual spinal canal area (RSCA-1) and residual spinal cord area (RSCA-2). (a) The area of the normal spinal canal. (b) The area of the narrow spinal canal. RSCA-1 or RSCA-2: S2/S1; RSCA-1 was evaluated by CT; and RSCA-2 was evaluated by MRI.

**Figure 2:** Illustration of the procedures of thoracic extensive laminoplasty (TELP) in a coronal view. (a) The thoracic spine with ossified ligamentum flavum (OLF in brown color). (b) Excision of the spinous process and portion of the lamina (not shown in the picture). (c) Bilateral grooves were made by grinding with a drill, and the lamina was isolated bilaterally. (d, e) Lifting the lamina (OLF in brown color) by towel forceps. (f) Fixation by arch plates and fusion with corticocancellous bone (not shown in the picture). (g) Intraoperative view of the TELP.

**Figure 3:** Illustration of the procedures of thoracic extensive laminoplasty (TELP) in a cross-section view. (a) The level of vertebra with TOLF. (b) Excision of the spinous process and portion of the lamina (not shown in the picture). (c) Bilateral grooves were made by grinding with a drill, and the lamina was isolated bilaterally. (d) Lifting the lamina by towel forceps. (e) Fixation by arch plates and fusion with corticocancellous bone (not shown in the picture).

**Figure 4:** A 45-years old patient with STOLF from T3 to T5 levels who received TELP. (a) Preoperative CT. (b) Preoperative MRI. (c, d) Postoperative standing anteroposterior X-ray at final follow-up. (e) Postoperative MRI at final follow-up. (f) Postoperative CT at final follow-up. (g) Postoperative three-dimensional CT reconstruction at final follow-up.

**Figure 5:** A 49-year-old patient with STOLF from T9 to T11 levels who received laminectomy. (a, b) Preoperative standing anteroposterior X-ray. (c) Preoperative CT. (d) Preoperative MRI. (e, f) Postoperative standing anteroposterior X-ray at final follow-up. (g, h) Postoperative MRI at final follow-up.

**Table 1:** Demographic characteristics (mean ± SD or *n*).

Item	G1	G2	*p* value
Sex, *n*	Male: 35	Male: 39	0.686
	Female: 24	Female: 23	
Age, years old	52.2 ± 4.7	51.8 ± 7.3	0.722
BMI, kg/m^2^	24.1 ± 2.6	23.7 ± 3.2	0.453
Symptom, *n* (%)			
LB numbness	42 (71.2)	46 (74.2)	0.710
LB spastic paraparesis	28 (47.5)	33 (53.2)	0.526
LB sensory deficits	49 (83.1)	51 (82.3)	0.908
Gait instability	26 (44.1)	29 (46.8)	0.765
Urinary sphincter dysfunction	18 (30.5)	22 (35.5)	0.561
Blood loss, ml	273.8 ± 31.7	281.4 ± 35.8	0.220
Operating room time, hours	3.5 ± 1.8	3.8 ± 1.6	0.334
Follow-up time, months	19.4 ± 2.1	18.9 ± 2.8	0.271
Dural laceration, *n*	0	17	——
Cerebrospinal fluid leakage, *n*	0	17	——

BMI: body mass index; LB: lower limbs.

**Table 2:** Image evaluation (mean ± SD or *n*).

Item	G1	G2	*p* value
Single level, *n*	10	15	0.325
≥2 levels, *n*	49	47	
DO or DA, *n*	50	52	0.895
RSCA-1			
Preoperation, %	37.9 ± 2.5	38.1 ± 3.2	0.703
Postoperation, %	78.2 ± 5.3	78.1 ± 4.8	0.913
*p* value	<0.0001	<0.0001	——
Improvement, %	40.3 ± 3.9	40.0 ± 4.1	0.681
RSCA-2			
Preoperation, %	37.2 ± 2.8	37.6 ± 2.6	0.417
Postoperation, %	79.4 ± 4.4	78.8 ± 3.9	0.428
*p* value	<0.0001	<0.0001	——
Improvement, %	42.2 ± 3.3	41.2 ± 2.9	0.079

Postoperation: postoperation at final follow-up. DO or DA: dural ossification or dural adhesion.

**Table 3:** Neurological evaluation based on mJOA (mean ± SD or *n*).

Item	G1	G2	*p* value
Preoperation	4.2 ± 1.4	4.3 ± 1.7	0.725
Postoperation	8.1 ± 1.9	7.9 ± 1.6	0.532
*p* value	<0.0001	<0.0001	——
≥50% *^Δ^*	31	18	0.008
<50% *^Δ^*	28	44	
OR (95% CI)	2.706 (1.279~5.727)		——

*^Δ^*Recovery rate. Postoperation: postoperation at final follow-up.

**Table 4:** HRQOL of the patients based on SF-36 (mean ± SD or *n*).

Item	PF		BP		GH		RHT	
	G1	G2	G1	G2	G1	G2	G1	G2
Pre	31.2 ± 11.4	31.7 ± 12.1	52.9 ± 11.7	53.1 ± 10.8	37.4 ± 13.9	37.2 ± 10.7	28.9 ± 8.7	28.2 ± 9.5
Post	71.6 ± 13.9	64.8 ± 11.7	80.6 ± 9.4	74.3 ± 7.1	73.4 ± 16.5	66.2 ± 12.2	70.7 ± 11.1	66.4 ± 10.9
P1 (G1/G2)	Pre: 0.816		Pre: 0.922		Pre: 0.268		Pre: 0.674	
	Post: 0.004		Post: <0.0001		Post: 0.007		Post: 0.034	
P2 (pre/post)	G1: <0.0001		G1: <0.0001		G1: <0.0001		G1: <0.0001	
	G2: <0.0001		G2: <0.0001		G2: <0.0001		G2: <0.0001	
	T/F	T/F	T/F	T/F	T/F	T/F	T/F	T/F
≥50%*^Δ^*	23/11	10/15	28/11	13/9	26/12	12/13	22/12	11/14
<50%*^Δ^*	8/17	20/17	3/17	17/23	5/16	18/19	9/16	19/18
*p* value	0.007	0.277	<0.0001	0.211	0.001	0.960	0.029	0.570
OR	4.443	—	14.424	—	6.933	—	3.259	—
(95% CI)	(1.471~13.423)	—	(3.516~59.181)	—	(2.057~23.368)	—	(1.109~9.576)	—

PF: physical functioning; BP: bodily pain; GH: general health; RHT: reported health transition; Pre: preoperation; Post: postoperation at final follow-up; T: tuberous type of STOLF; F: fused-type PF STOLF; *^Δ^*recovery rate.

## Data Availability

All the data associated with this article is deposited in the table part (Tables 1to 4).
